# The Effects of Ticagrelor Combined with Tirofiban on Coagulation Function, Serum Myocardial Injury Markers, and Inflammatory Factor Levels in Patients with Acute Myocardial Infarction after Percutaneous Coronary Intervention

**DOI:** 10.1155/2022/4217270

**Published:** 2022-04-28

**Authors:** Fang Li, Shuhui Wang, Lei Wang, Feng Liu, Zhen Meng, Jia Liu

**Affiliations:** ^1^Department of Clinical Laboratory, Yantaishan Hospital, Yantai 264000, Shandong Province, China; ^2^Department of Clinical Laboratory, The Affiliated Qingdao Central Hospital of Qingdao University, The Second Affiliated Hospital of Medical College of Qingdao University, Qingdao 266042, Shandong Province, China; ^3^ICU, The Affiliated Qingdao Central Hospital of Qingdao University, The Second Affiliated Hospital of Medical College of Qingdao University, Qingdao 266042, Shandong Province, China; ^4^Department of Spine Surgery, Zhangqiu District People's Hospital, Jinan 250200, Shandong Province, China; ^5^Department of Ultrasound, Zhangqiu District People's Hospital, Jinan 250200, Shandong Province, China; ^6^ICU, Yantai Yuhuangding Hospital Affiliated to Qingdao University, Yantai 264000, Shandong Province, China

## Abstract

**Background:**

Acute myocardial infarction (AMI) refers to the acute necrosis of part of the myocardium caused by persistent and severe myocardial ischemia. This study is aimed at investigating the efficacy of tirofiban combined with ticagrelor in AMI patients after percutaneous coronary intervention (PCI) and its effects on plasma activated partial thromboplastin time (APTT), fibrinogen (FIB), D-dimer (D-D) levels, myocardial injury markers, and inflammatory factors.

**Methods:**

68 AMI patients with AMI who received PCI were divided into control group and observation group (n =34) according to postoperative treatment methods. Both groups received ticagrelor tablets (90 mg). The observation group was additionally given tirofiban (10 *μ*g/kg). APTT, FIB, D-D, serum myoglobin (MB), cardiac troponin I (cTnI), serum C-reactive protein (CRP), tumor necrosis factor-*α* (TNF-*α*), and IL-6, myeloperoxidase (MPO) levels and the peak time in both groups were detected. The incidence of cardiovascular events and drug safety were compared.

**Results:**

After treatment, APTT was increased, and FIB and D-D levels were decreased in both groups. After treatment, the APTT in the observation group was longer, and FIB and D-D levels were lower than those in the control group. The peak time of serum MB and cTnI in the observation group was earlier than that in the control group. The levels of serum MB and cTnI in the observation group were lower than those in the control group. After treatment, serum CRP, TNF-*α*, IL-6, and MPO levels were decreased. And the incidence of cardiovascular events was reduced.

**Conclusion:**

Tirofiban combined with ticagrelor can improve coagulation function, protect myocardium, relieve inflammation, and reduce the risk of cardiovascular events in patients with AMI after PCI.

## 1. Introduction

Acute myocardial infarction (AMI) is a common cardiovascular emergency [1]. With the improvement of living standards, the number of patients with cardiovascular disease has also increased rapidly. Epidemiological surveys show that AMI has become the main cause of death and disability in Western countries. According to the World Health Organization (WHO), by 2020, AMI will rise from the fifth leading cause of death to the first globally [2]. AMI is an acute and critical cardiovascular disease caused by acute and persistent ischemia and hypoxia of coronary artery. The disease progresses rapidly with high morbidity and mortality [3].

The treatment of AMI has changed dramatically over the past two decades. Medications that improve prognosis are used regulated, including antiplatelet drugs [4], beta-blockers [5], angiotensin-converting enzyme inhibitors (ACEI) [6], and statins [7]. In addition, early reperfusion therapy including emergency interventional therapy (percutaneous coronary intervention (PCI)) and thrombolytic therapy is also becoming more and more mature [8]. Infarct-related blood vessels can be opened in the shortest time, greatly improving the prognosis of AMI and reducing mortality. Revascularization of infarct-related arteries (RA) by PCI can restore coronary blood flow in a timely and effective manner. This not only reduces the extent of myocardial ischemia and rescues dying myocardium but also improves the prognosis of patients [9–12]. However, during PCI, the thrombus may fall off again or form stent thrombosis, leading to distal microvascular embolism, thereby affecting the recovery of coronary blood flow and tissue-level perfusion. Therefore, it is particularly important to strengthen anticoagulation and antiplatelet therapy during surgery [13–15].

Ticagrelor, a selective adenosine diphosphate (ADP) receptor antagonist, is often used in combination with aspirin to reduce the risk of thrombotic cardiovascular events in patients after PCI [16–19]. The tirofiban platelet glycoprotein IIb/IIIa receptor is highly selective and specific and can compete with fibrinogen for platelet binding. Tirofiban exerts its antiplatelet aggregation effect by blocking the platelet aggregation channel [20, 21]. Previous studies have found [22, 23] that tirofiban combined with ticagrelor can effectively improve myocardial microcirculation in patients with PCI, and the efficacy is better than that of single drug. However, the dosage of tirofiban during PC1 surgery has a great influence on the incidence of adverse reactions such as bleeding [24]. Therefore, exploring the appropriate dosage of tirofiban has positive clinical implications.

This study investigated the effect of ticagrelor combined with tirofiban on coagulation function, serum myocardial injury markers, and inflammatory factor levels in patients with AMI after PCI.

## 2. Materials and Methods

### 2.1. Patients

From January 2020 to June 2021, a total of 68 patients with AMI who received PCI in Yantaishan Hospital were divided into control group and observation group (*n* = 34) according to postoperative treatment. There was no significant difference in general data between the two groups (*P* > 0.05, Table 1). The research protocol was reviewed and approved by the Medical Ethics Committee of Yantaishan Hospital. All patients or their families were informed and signed informed consent.

### 2.2. Inclusion and Exclusion Criteria

Inclusion criteria are as follows: (1) The age range is between 18 and 80 years old. (2) All patients underwent myocardial contrast echocardiography after admission. (3) All patients received PCI successfully after admission.

Exclusion criteria are as follows: (1) There is a recent history of active bleeding, such as active peptic ulcer; (2) hemodynamic instability; (3) coagulation dysfunction; (4) those who have received antiplatelet drugs and anticoagulant drugs in the past; (5) liver and renal dysfunction; (6) previous PCI, coronary artery bypass grafting (CABG), and angiography showed coronary collateral circulation grade 1-3 (Rentrop's classification); and (7) patients with immune system diseases, infections, malignant tumors, pregnant and breastfeeding women.

### 2.3. Treatment

After diagnosis, blood pressure, blood lipids, and blood sugar were controlled in both groups. Atorvastatin calcium tablets (10 mg, 1 time/d) and isosorbide mononitrate tablets (20 mg, 2 times/d) were given. Oral aspirin (300 mg) and ticagrelor (180 mg) were administered before treatment.

The observation group was given aspirin (100 mg, once/day) and ticagrelor (90 mg, twice/day) after operation. During PCI, tirofiban (10 *μ*g/kg) was injected into the coronary artery after passing the lesion target. And the injection was completed within 3 minutes. Both groups were given dual antiplatelet oral therapy (aspirin 100 mg/d+ticagrelor 90 mg/d) after surgery. Both groups were followed up to 6 months postoperatively.

### 2.4. Cardiac Function Comparison

Cardiac function tests were performed using GE VIVID7 echocardiography. The cardiac function indexes at 1 week and 6 months after surgery included left ventricular ejection fraction (LVEF), left ventricular end-systolic volume (LVESV), and left ventricular end-diastolic volume (LVEDV).

### 2.5. Coagulation

Before and after treatment, 5 mL of fasting venous blood was drawn from patients. ACL-TOP-700 automatic blood coagulation analyzer was used to detect plasma activated partial thromboplastin time (APTT) and fibrinogen (FIB) levels by coagulation method. D-dimer (D-D) level was detected by enzyme-linked immunosorbent assay.

### 2.6. Myocardial Injury Marker Peak Time

The peak times of serum myoglobin (MB) and cardiac troponin I (cTnI) were compared between the two groups. 3 mL of peripheral venous blood was collected from the two groups at 0, 10, 14, 24, and 36 hours after operation, respectively. MB and cTnI were detected using an automatic immunofluorescence microplate reader (Azure Biosystems). The levels of MB and cTnI were detected by the double-antibody sandwich chemiluminescence method.

### 2.7. Inflammatory Factor

Before and after treatment, 5 mL of fasting venous blood was collected from all patients. After centrifugation at 3000 r/min for 10 min, it was stored in a -70°C refrigerator for testing. The detection instrument is Brocade BIOBASE 2001 automatic enzyme immunoassay analyzer. ELISA was used to detect the levels of IL-6, serum C-reactive protein (CRP), tumor necrosis factor-*α* (TNF-*α*), and myeloperoxidas (MPO).

### 2.8. Major Adverse Cardiovascular Events (MACEs)

Follow-up for 1 year, the occurrence of MACEs in the two groups, such as cardiac death, recurrent myocardial infarction, stent thrombosis, and target vessel reconstruction, was recorded.

### 2.9. Statistical Analysis

All experiments were repeated 3 times. The data were analyzed by SPSS22.0 statistical analysis software and expressed as $\bar{x}\pm s$. Differences were compared using ANOVA or Chi-square test. The *t*-test was used to compare data between the same groups. *P* < 0.05 indicated that the difference was statistically significant.

## 3. Results

### 3.1. Comparison of Cardiac Function between the Two Groups

The LVEF, LVEDD, and LVESD of the two groups were measured by GE VIVID7 echocardiography after PCI for 1 week. There was no significant difference in LVEF, LVEDV, and LVESV between the two groups before treatment (*P* > 0.05, Figure 1). The cardiac function indexes after treatment were better than those before treatment (*P* < 0.05, Figure 1). Compared with the control group, the levels of LVEDD and LVESD in the observation group were decreased, and the level of LVEF was increased (*P* < 0.05, Figure 1). After treatment, the improvement of cardiac function indexes in the observation group was better than that in the control group (*P* < 0.05, Figure 1).

### 3.2. Comparison of Coagulation Function between the Two Groups

Before treatment, there was no significant difference in plasma APTT, FIB, and D-D levels between the two groups (*P* > 0.05, Figure 2). After treatment, APTT was increased, and FIB and D-D levels were decreased in both groups (*P* < 0.05, Figure 2). After treatment, APTT in the observation group was increased, and the levels of FIB and D-D were lower than those in the control group (*P* < 0.05, Figure 2).

### 3.3. Comparison of the Peak Time of Myocardial Injury Markers between the Two Groups

Compared with the control group, the serum MB and cTnI peaks in the observation group were significantly decreased (*P* < 0.05, Figure 3). The levels of serum MB and cTnI in the observation group were lower than those in the control group (*P* < 0.05, Figure 3). The results suggest that ticagrelor combined with tirofiban can reduce serum cTnI and CK-MB levels, effectively improve myocardial ischemia, and exert myocardial protection.

### 3.4. Comparison of Inflammatory Factor Levels between Two Groups

Before treatment, there was no significant difference in the levels of serum inflammatory factors CRP, TNF-*α*, IL-6, and MPO between the two groups (*P* > 0.05, Figure 4). After treatment, serum CRP, TNF-*α*, IL-6, and MPO in both groups were decreased (*P* < 0.05, Figure 4). Compared with the control group, the levels of serum inflammatory factors CRP, TNF-*α*, IL-6, and MPO in the observation group were reduced (*P* < 0.05, Figure 4). These results suggest that the ability of ticagrelor combined with tirofiban to relieve inflammatory factors is higher than that of ticagrelor alone.

### 3.5. Comparison of the Incidence of MACE in the Two Groups of Patients

During the follow-up period after treatment, the incidence of MACE was 35.3% in the control group and 9.1% in the observation group. The total incidence of cardiovascular events in the observation group was lower than that in the control group (Table 2).

## 4. Discussion

PCI is the first choice for clinical treatment of AMI patients. However, it needs to be used in conjunction with antiplatelet drugs to prevent thrombus from falling off or the formation of stent thrombosis, which affects the efficacy [14, 15]. Aspirin and ticagrelor are commonly used antiplatelet drugs in clinical practice. Aspirin and ticagrelor can prevent platelet aggregation by blocking the TXA pathway and the P2Y12ADP receptor pathway but have no significant effect on the final pathway of platelet aggregation [25]. It has been shown that [26] platelet glycoprotein IIb/IIIA receptors play a key role in the process of platelet aggregation. The final pathway can be blocked with IIb/IIIA receptor antagonists. Tirofiban, a receptor antagonist with strong antiplatelet effect, can be injected directly into the coronary arteries. Tirofiban is highly specific and can act on platelets rapidly, directly, and reversibly to inhibit thrombosis. This study showed that tirofiban combined with ticagrelor had a more significant effect on improving cTFC and coronary recanalization rate in patients with PCI than ticagrelor alone. Tirofiban combined with ticagrelor can prevent and reduce thrombosis and improve coronary blood flow in patients after PCI.

MB and cTnI are markers of myocardial injury, and their serum levels are proportional to the degree of myocardial damage [27]. During recanalization after PCI, MB and cTnI enter the blood with the recovery of blood flow, resulting in a peak migration. Therefore, the peak time of serum MB and cTnI is of great significance for monitoring. This study showed that tirofiban could advance the peak time of serum MB and cTnI and achieve coronary reperfusion as soon as possible. It can effectively treat infarcted myocardial tissue and reduce the degree of myocardial damage. This is related to the potent antiplatelet and endothelial protective effects of tirofiban. Tirofiban can not only block the final pathway of platelet aggregation by antagonizing GPIIb/IIIA receptors but also inhibit the release of serotonin and thromboxane A2 from platelets, thereby inhibiting vasoconstriction and maintaining the relaxation response of distal coronary vessels. In addition, tirofiban can also regulate vascular endothelial function by increasing endogenous NO. Therefore, tirofiban has a good effect on improving coronary blood flow and can advance the peak time of serum myocardial injury markers.

The occurrence of AMI and PCI will aggravate the inflammatory response of patients, manifested as increased serum inflammatory factor levels. Persistent inflammatory responses exacerbate blood hypercoagulation and vascular endothelial damage and increase the risk of disease progression and recurrence. CRP is an acute phase response protein and a nonspecific marker of inflammation and tissue damage. Its serum level rises rapidly when acute inflammation and tissue damage occurs. And the increase rate of CRP was positively correlated with the degree of damage prevention. TNF-*α* has immune and inflammatory regulatory effects. High concentrations of TNF-*α* can reduce myocardial contractile function and induce myocardial dysfunction and myocardial inflammation. MPO, a leukocyte-derived enzyme, is an early marker of acute coronary syndrome. Its serum levels were positively correlated with inflammatory activity. High levels of MPO exacerbate arteriosclerosis and promote disease progression [28].

This study investigated the efficacy of ticagrelor combined with tirofiban in the treatment of AMI patients with PCI. Compared with ticagrelor alone, the levels of FIB, D-D, serum MB, cTnI, serum CRP, TNF-*α*, IL-6, MPO, and the incidence of cardiovascular events were significantly reduced in the ticagrelor combined with tirofiban group. The peak time of serum MB and cTnI was earlier, and the APTT was prolonged in the ticagrelor combined with tirofiban group. However, the sample size of this study is small. We still need to expand the sample size in the future to further verify our conclusions.

## 5. Conclusion

In conclusion, tirofiban combined with ticagrelor can effectively improve coronary blood flow recanalization rate, improve myocardial injury, and reduce inflammatory response in AMI patients with PCI. And it can also reduce the incidence of cardiovascular events, with good safety.

## Figures and Tables

**Figure 1:** Comparison of LVEF, LVEDD, and LVESD before and after treatment in the two groups (*n* = 34). ^∗^*P* < 0.05, compared with before treatment; ^#^*P* < 0.05, compared with the control group.

**Figure 2:** Comparison of plasma APTT, FIB, and D-D levels before and after treatment in the two groups (*n* = 34). ^∗^*P* < 0.05, compared with before treatment; ^#^*P* < 0.05, compared with the control group.

**Figure 3:** Comparison of myocardial injury markers between the two groups of patients (*n* = 34). ^#^*P* < 0.05, compared with the control group.

**Figure 4:** Comparison of inflammatory factor levels before and after treatment in two groups of patients (*n* = 34). ^∗^*P* < 0.05, compared with before treatment; ^#^*P* < 0.05, compared with the control group.

**Table 1:** Comparison of baseline characteristics of patients in the two groups.

Features	Control group (*n* = 34)	Observation group (*n* = 33)	*t*/*χ*^2^	*P*
Gender			0.008	0.93
Male	22 (64.7%)	21 (63.6%)		
Female	12 (35.3%)	12 (36.4%)		
Age (year)	56.76 ± 8.02	56.82 ± 7.96	0.03	0.98
Complication				
Hypertension	21 (61.8%)	23 (69.7%)	0.47	0.49
Hyperlipidemia	25 (73.5%)	27 (81.2%)	0.66	0.42
Diabetes	7 (20.6%)	8 (24.2%)	0.13	0.72

**Table 2:** Comparison of major cardiovascular events between the two groups of patients (cases (%)).

Group	Heart failure	Malignant arrhythmia	Cardiogenic shock	Reinfarction	Total
Control group	2 (5.9%)	3 (8.8%)	3 (8.8%)	4 (11.8%)	12 (35.3%)
Observation group	1 (3.0%)	1 (3.0%)	0 (0.0%)	1 (3.0%)	3 (9.1%)

## Data Availability

The data used to support the findings of this study are available from the corresponding author upon request.

## References

[1] Weir R. A., McMurray J. J., Velazquez E. J. (2006). Epidemiology of heart failure and left ventricular systolic dysfunction after acute myocardial infarction: prevalence, clinical characteristics, and prognostic importance. *The American Journal of Cardiology*.

[2] Lopez A. D., Murray C. C. (1998). The global burden of disease, 1990-2020. *Nature Medicine*.

[3] Desai N. R., Kennedy K. F., Cohen D. J. (2017). Contemporary risk model for inhospital major bleeding for patients with acute myocardial infarction: the acute coronary treatment and intervention outcomes network (ACTION) registry®-Get With The Guidelines (GWTG)®. *American Heart Journal*.

[4] Yusuf S., Zhao F., Mehta S. R. (2001). Effects of clopidogrel in addition to aspirin in patients with acute coronary syndromes without ST-segment elevation. *The New England Journal of Medicine*.

[5] ISIS-1 (First International Study of Infarct Survival) Collaborative Group (1986). Randomised trial of intravenous atenolol among 16,027 cases of suspected acute myocardial infarction: ISIS‐1. *Lancet*.

[6] ACE Inhibitor Myocardial Infarction Collaborative Group (1998). Indications for ACE inhibitors in the early treatment of acute myocardial infarction: systematic overview of individual data from 100, 000 patients in randomized trials. *Circulation*.

[7] Long-Term Intervention with Pravastatin in Ischaemic Disease Study G (1998). Prevention of cardiovascular events and death with pravastatin in patients with coronary heart disease and a broad range of initial cholesterol levels. *The New England Journal of Medicine*.

[8] Faxon D. P. (2005). Coronary interventions and their impact on post myocardial infarction survival. *Clinical Cardiology*.

[9] Eagle K. A., Nallamothu B. K., Mehta R. H. (2008). Trends in acute reperfusion therapy for ST-segment elevation myocardial infarction from 1999 to 2006: we are getting better but we have got a long way to go. *European Heart Journal*.

[10] Gibson C. M., Pride Y. B., Frederick P. D. (2008). Trends in reperfusion strategies, door-to-needle and door-to-balloon times, and in-hospital mortality among patients with ST-segment elevation myocardial infarction enrolled in the National Registry of Myocardial Infarction from 1990 to 2006. *American Heart Journal*.

[11] Remkes W. S., Somi S., Roolvink V. (2014). Direct drug-eluting stenting to reduce stent restenosis: a randomized comparison of direct stent implantation to conventional stenting with pre- dilation or provisional stenting in elective PCI patients. *JACC. Cardiovascular Interventions*.

[12] McCormick L. M., Brown A. J., Ring L. S. (2014). Direct stenting is an independent predictor of improved survival in patients undergoing primary percutaneous coronary intervention for ST elevation myocardial infarction. *European Heart Journal Acute Cardiovascular Care*.

[13] Choi J. H., Cho J. R., Park S. M. (2017). Sarpogrelate based triple antiplatelet therapy improved left ventricular systolic function in acute myocardial infarction: retrospective study. *Yonsei Medical Journal*.

[14] Esposito M. L., Zhang Y., Qiao X. (2018). Left ventricular unloading before reperfusion promotes functional recovery after acute myocardial infarction. *Journal of the American College of Cardiology*.

[15] Thiele H., Akin I., Sandri M. (2017). PCI strategies in patients with acute myocardial infarction and cardiogenic shock. *The New England Journal of Medicine*.

[16] Kristensen S. D., Würtz M., Grove E. L. (2012). Contemporary use of glycoprotein IIb/IIIa inhibitors. *Thrombosis and Haemostasis*.

[17] Grove E. L., Kristensen S. D. (2009). Update on oral antiplatelet therapy: principles, problems and promises. *Future Cardiology*.

[18] Levine G. N., Bates E. R., Blankenship J. C. (2011). 2011 ACCF/AHA/SCAI guideline for percutaneous coronary intervention: a report of the American College of Cardiology Foundation/American Heart Association task force on practice guidelines and the Society for Cardiovascular Angiography and Interventions. *Circulation*.

[19] Amsterdam E. A., Wenger N. K., Brindis R. G. (2014). 2014 AHA/ACC guideline for the management of patients with non-ST-elevation acute coronary syndromes: a report of the American College of Cardiology/American Heart Association task force on practice guidelines. *Journal of the American College of Cardiology*.

[20] Kajiwara M., Tanaka A., Kawasaki T. (2017). Safety and efficacy of liraglutide treatment in Japanese type 2 diabetes patients after acute myocardial infarction: a non-randomized interventional pilot trial. *Journal of Cardiology*.

[21] Yu H., Ma L., Feng K., Chen H., Hu H. (2017). Clinical application of optical coherence tomography in patients with non-ST-elevation acute coronary syndrome combined with intermediate lesions. *The Heart Surgery Forum*.

[22] Storey R. F., Angiolillo D. J., Patil S. B. (2010). Inhibitory effects of ticagrelor compared with clopidogrel on platelet function in patients with acute coronary syndromes: the PLATO (PLATelet inhibition and patient Outcomes) PLATELET substudy. *Journal of the American College of Cardiology*.

[23] Heusch G., Kleinbongard P., Böse D. (2009). Coronary microembolization: from bedside to bench and back to bedside. *Circulation*.

[24] Wang H., Feng M. (2020). Influences of different dose of tirofiban for acute ST elevation myocardial infarction patients underwent percutaneous coronary intervention. *Medicine*.

[25] Kobzar G., Mardla V., Samel N. (2017). Glucose impairs aspirin inhibition in platelets through a NAD(P)H oxidase signaling pathway. *Prostaglandins & Other Lipid Mediators*.

[26] Begkas D., Chatzopoulos S. T., Touzopoulos P., Balanika A., Pastroudis A. (2020). Ultrasound-guided platelet-rich plasma application versus corticosteroid injections for the treatment of greater trochanteric pain syndrome: a prospective controlled randomized comparative clinical study. *Cureus*.

[27] Iakovou I., Mintz G. S., Dangas G. (2003). Increased CK-MB release is a “trade-off” for optimal stent implantation: an intravascular ultrasound study. *Journal of the American College of Cardiology*.

[28] Cavusoglu E., Ruwende C., Eng C. (2007). Usefulness of baseline plasma myeloperoxidase levels as an independent predictor of myocardial infarction at two years in patients presenting with acute coronary syndrome. *The American Journal of Cardiology*.

